The article "Seizure freedom without seizure medication following stereoelectroencephalography implantation: a case report of drug-resistant post-traumatic epilepsy" was retracted in 2024. Reason: duplicate publication.

# Seizure freedom without seizure medication following stereoelectroencephalography implantation: a case report of drug-resistant post-traumatic epilepsy

**DOI:** 10.3389/fneur.2024.1391439

**Published:** 2024-04-25

**Authors:** Alexander Tran, Marjorie Bunch

**Affiliations:** Albany Medical Center, Albany, NY, United States

**Keywords:** stereoelectroencephalography, drug-resistant epilepsy, intracranial electrodes, microlesion effects, seizure remission

## Abstract

Achieving seizure freedom following failure of several antiseizure medications (ASMs) is rare, with the likelihood of achieving further control decreasing with each successive ASM trial. When cases of drug-resistant epilepsy arise, a diagnostic procedure known as stereoelectroencephalography (sEEG) can be used to identify epileptogenic zones (EZ) within the brain. After localization of these zones, they can be targeted for future surgical intervention. Here, we describe a case of complete seizure freedom off medication after sEEG without resection or other therapeutic intervention. In 2017, a 36-year-old right-handed male presented with drug-resistant epilepsy stemming from prior traumatic brain injury. Due to ongoing seizures, in 2020 a robotic-assisted sEEG electrode placement procedure was employed to localize the seizure onset zone. During sEEG monitoring, a single event was captured where the patient had dysarthric speech, left arm dystonic flexion, and difficulty responding to questioning. Notably, this event had no sEEG correlate, suggesting seizure occurrence in a region not monitored by implanted electrodes, which prompted the placement of scalp electrodes following this event. However, no further clinical events consistent with seizure were provoked through the remainder of recording. Following the 13-day admission, the patient chose to self-discontinue all seizure medications and has remained seizure free as of October 2023, more than 3.5 years later. While sEEG is considered a relatively safe procedure for seizure localization in drug resistant epilepsy, the possibility of microlesions created by sEEG depth electrodes remains largely unexplored. Further evaluation should be performed into potential tissue injury produced by depth electrode insertion.

## Introduction

Obtaining seizure freedom after failure of multiple antiseizure medications (ASMs) is uncommon, with additional seizure control diminishing with successive ASM trials (1). In cases of drug-resistant epilepsy, stereoelectroencephalography (sEEG) is a diagnostic procedure used in the evaluation and targeting of potential epileptogenic zones (EZ) for future surgical resection (2). Typically, anywhere from 6 to 15 depth electrodes are placed in areas of the brain where EZ are suspected based on presurgical testing including video EEG and MRI findings (3). Advancements in robotic technology such as robotic stereotactic assistance have allowed the implantation of multiple intracranial electrodes without the assistance of a frame-based technique, resulting in more accurate targeting of deep cortical tissue, and decreased operating time (3). Despite being primarily a monitoring procedure, sEEG has shown potential in rare instances to induce seizure remission upon removal of depth electrodes (4). Here, we describe a patient who underwent sEEG monitoring with complete remission of habitual seizures upon initial implantation of depth electrodes who remained seizure free for more than 3 years off all seizure medications.

## Case report

Patient initially presented in 2017 as a 36-year-old male with focal epilepsy related to remote traumatic brain injury. In 1998, the patient reported a convulsive episode after being an unrestrained passenger in a motor vehicle accident with traumatic head injury requiring shunt, resulting in residual left leg weakness and cognitive impairment. The patient was involved in another motor vehicle accident in 2001, with another reported head trauma but no documented seizure activity. An additional poorly described seizure was reported while incarcerated in 2007, followed by an extended period of seizure freedom until June 2016. From then on, the patient suffered recurrent seizures, occurring once every 1–2 weeks, sometimes in clusters and often during sleep or upon awakening. Typical seizure semiology was described as behavioral arrest, oral automatisms or automatic speech, head and eye deviation to the left, sometimes preceded by olfactory aura of smoke. Postictally, he reported a left hemiparesis. Neurological examination at baseline was pertinent for left greater than right lower extremity spasticity, mild weakness in the left leg, and bilateral ankle clonus. Over several years, multiple ASMs including levetiracetam 750 mg twice daily, gabapentin 800 mg four times daily, lamotrigine 250 mg twice daily, topiramate 150 mg twice daily, clobazam 20 mg twice daily, and perampanel 4 mg daily failed to resolve seizures.

Due to drug resistant seizures, the patient underwent a three-day long video EEG monitoring session, during which a total of 10 right temporal regional focal onset electrographic seizures were captured (onset Figure 1). Among these seizures, nine exhibited a distinct clinical correlate with right-hand or bimanual automatisms, as well as oral automatisms, with most progressing into bilateral tonic–clonic seizures. The admission also captured presumed surface negative focal aware seizures with delayed pupillary dilatation and a sensation of being “outside of oneself.” Interictally, the EEG demonstrated mild intermittent polymorphic right temporal slowing along with occasional right temporal sharp and spike wave discharges consistent with focal cerebral dysfunction and seizure risk (Figure 2).

**Figure 1:** Ictal EEG from 3-day phase 1 session. EEG results showing seizure onset modified bipolar montage with sub temporal chains, sensitivity 7 microvolts/cm, high cut: 15 Hz, low cut: 1.0 Hz. At 21:12:12 the patient awoke and put right hand over his face. Electrographic onset noted at 21:12:25 with rhythmic theta in the right temporal and subtemporal chains preceded oral automatisms (marked).

**Figure 2:** Interictal EEG of right temporal sharp waves. EEG results showing right temporal sharp waves with modified bipolar montage with sub temporal chains, sensitivity 7 microvolts/cm, high cut: 70 Hz, low cut: 1.0 Hz.

Workup also included a 2019 MRI of the brain with intravenous contrast, showing patchy areas of FLAIR hyperintensities within the bilateral anterior frontal periventricular white matter extending along the forceps minor (Figure 3). A linear area of encephalomalacia with surrounding gliosis in the anterior right frontal lobe was consistent with previous catheterization. Additional areas of encephalomalacia and gliosis were seen in the medial right frontoparietal junction as well as in the bilateral periventricular white matter. Possible hemosiderin staining was noted in the medial right frontoparietal junction. Severe thinning of the posterior body of the corpus callosum and mild cerebral volume loss were also identified. Neuropsychological testing in the same year showed mild deficits on visual tasks as well as left hand fine motor dexterity, both deficits consistent with right hemisphere dysfunction. PET-CT scan was negative.

**Figure 3:** Abnormal MRI with IV Contrast. 2019 MRI brain FLAIR images utilizing a 3 T magnet with intravenous contrast show multiple zones of encephalomalacia due to prior traumatic brain injury and right ventricular catheterization.

In 2020 the patient underwent a robotic assisted right hemispheric stereo EEG electrode placement procedure without complication, utilizing a robotic surgical assistant. This involved the positioning of 11 electrodes targeting specific anatomic locations to localize the seizure onset zone (Figure 4). Initially, hypothesis for implantation favored mesial temporal onset due to observed auras; however, concerns arose regarding the possibility of multiple seizure foci and potential extra-temporal onset. The final implantation strategy aimed to target limbic structures, regions capable of mimicking temporal semiology, and to sample areas exhibiting cortical scarring as identified on MRI. These depth electrodes (0.8 mm diameter, 5 mm between contacts) included: parietal lesion (10 contacts), mesial parietal lesion (8 contacts), anterior cingulate (12 contacts), middle cingulate (12 contacts), posterior cingulate (14 contacts), frontopolar (14 contacts), posterior periinsular (8 contacts), hippocampal tail (10 contacts), basal frontal (16 contacts), uncus (12 contacts), and hippocampal head (12 contacts). A post-operative head CT confirmed placement of electrodes and did not identify any areas of hemorrhage or hematoma. The patient underwent video sEEG monitoring for 13 days.

**Figure 4:** Final placement of sEEG electrodes under X-ray. Post implantation X-ray showing right hemisphere depth electrode placement.

Provocation of seizures was attempted with medication taper and cessation of seizure medications (clobazam, lamotrigine, gabapentin), sleep deprivation, and two challenges of intravenous lorazepam followed by flumazenil. Interictal sEEG findings demonstrated spikes from the hippocampus and the posterior cingulate gyrus. A single clinical event was captured the morning after implantation where the patient wiped his right hand on his mouth, then had dysarthric speech, left arm dystonic flexion, and difficulty responding to questioning. This event had no sEEG correlate, suggesting seizure occurrence in a region not monitored by sEEG, prompting the placement of scalp electrodes following this event. This event did not resemble his habitual seizures. No further clinical events consistent with seizure were provoked through the remainder of recording and no electrographic seizures were captured. Head CT performed after electrode removal demonstrated numerous small right sided foci of pneumocephalus without evidence of intracranial hemorrhage. Following the 13-day admission, the patient chose not to resume any seizure medications despite counseling otherwise and remains seizure free 3.5 years after sEEG, confirmed by his wife. Most recent head CT in 2023 showed no additional areas of encephalomalacia.

## Discussion

This case describes a man with post-traumatic drug resistant epilepsy who has had no typical seizures for more than 3 years following stereo EEG implantation despite complete medication cessation. One single atypical event during invasive monitoring suggestive of an acute symptomatic seizure was captured on sEEG suggesting a focal seizure limited to unsampled cortex. A non-epileptic event could not be excluded. Potential causes of an atypical seizure include direct cortical irritation caused by electrode insertion, hemorrhage/hematoma, edema, or pneumocephalus with the effects of anesthesia withdrawal possibly contributing. Another possibility is that the clinical symptoms were the result of focal vascular changes related to local injury.

The abrupt cessation of all seizures without seizure medication after intracranial monitoring suggests epilepsy remission due to effects of sEEG implantation, however this report is limited as there is no objective evidence to confirm causality. A post-operative MRI was not performed, which could have shown new areas of encephalomalacia or hemosiderin deposition to support this association. Likewise, no further EEG studies were performed to assess for ongoing cortical irritability.

While the literature acknowledges instances of sEEG monitoring resulting in seizure remission, these occurrences are particularly rare (5), with a previous study of epilepsy patients observing 0.5% remission rate following intracranial electrode placement. A previous case series described 3 patients with seizure remission following sEEG, however, these cases reported multiple seizures captured during the monitoring period (6), proving accurate targeting of the seizure onset zone with electrodes and suggesting the lesioning effect was not upon initial implantation but rather because of depth electrode removal or other delayed effects. In addition, none of the prior cases reported complete discontinuation of seizure medications. Our case is also notable in that the presumed etiology of epilepsy was trauma, and preimplantation imaging demonstrated multiple areas of injury. It is therefore more surprising that a small lesion was adequate to disrupt the epileptogenic network so completely to result in seizure freedom off medication. In support of this theory, evidence suggests minimally invasive techniques such as radiofrequency thermocoagulation can adequately disrupt widespread pathological networks in lesions such as periventricular nodular heterotopia resulting in seizure freedom (7).

Intracranial electrode placement resulting in microlesion effects has been documented in multiple cases regarding Parkinson’s disease (8). A systematic meta-analysis of sEEG complications found that sEEG displays a low complication rate of 1.3% in comparison to other methods of invasive monitoring (2). Further investigation revealed that most of these complications come from hemorrhage with a pooled prevalence of 1% (2). A unique study that evaluated the neuropsychological impact of hippocampal depth electrodes placed along the longitudinal axis in the language dominant hemisphere suggested possible verbal memory deterioration (9). While this study was limited by power and other design flaws, it suggested that further evaluation for potential effects of electrode insertion may be warranted to better characterize network impacts.

This case adds to the growing literature that suggests potential for clinically significant consequences from depth electrode insertion. The implications are that while sEEG is overall relatively safe and can be useful for evaluation of drug resistant epilepsy, there remains a largely unexplored possibility of microlesion effects, which could result in either beneficial or harmful sequelae for patients. Our recommendation is for ongoing investigations into the long-term consequences of depth electrode implantation with attention to both localized effects as well as changes to epileptic and cognitive networks.

## Data availability statement

The original contributions presented in the study are included in the article/supplementary material, further inquiries can be directed to the corresponding author.

## Author contributions

AT: Writing – original draft, Writing – review & editing. MB: Writing – review & editing.

## References

[1] ChenZ.BrodieM.J.LiewD.KwanP., (2018). Treatment outcomes in patients with newly diagnosed epilepsy treated with established and new antiepileptic drugs: a 30-year longitudinal cohort study. JAMA Neurol 75, 279–286. doi: 10.1001/jamaneurol.2017.394929279892 PMC5885858

[2] MullinJPShriverMAlomarSNajmIBulacioJChauvelP. Is sEEG safe? A systematic review and meta-analysis of stereo-electroencephalography-related complications. Epilepsia. (2016) 57:386–401. doi: 10.1111/epi.13298, PMID: 26899389

[3] KhooHMHallJADubeauFTaniNOshinoSFujitaY. Technical aspects of sEEG and its interpretation in the delineation of the epileptogenic zone. Neurol Med Chir. (2020) 60:565–80. doi: 10.2176/nmc.st.2020-0176PMC780370333162469

[4] KatariwalaNMBakayRAPennellPBOlsonLDHenryTREpsteinCM. Remission of intractable partial epilepsy following implantation of intracranial electrodes. Neurology. (2001) 57:1505–7. doi: 10.1212/WNL.57.8.1505, PMID: 11673602

[5] OjemannLMDodrillCB. Natural history of drug resistant seizures: clinical aspects. Epilepsy Res Suppl. (1992) 5:13–7. PMID: 1418442

[6] KaurM.SzaflarskiJ.P.Ver HoefL.PatiS.RileyK.O.JaisaniZ., (2019). Long-term seizure freedom following intracranial sEEG monitoring: therapeutic benefit of a diagnostic technique. Epilepsy Behav Rep 12,:100345, doi: 10.1016/j.ebr.2019.10034531799508 PMC6883308

[7] MirandolaLMaiRFFrancioneSPellicciaVGozzoFSartoriI. Stereo-EEG: diagnostic and therapeutic tool for periventricular nodular heterotopia epilepsies. Epilepsia. (2017) 58:1962–71. doi: 10.1111/epi.13895, PMID: 28880999

[8] TykockiTNaumanPKoziaraHMandatT. Microlesion effect as a predictor of the effectiveness of subthalamic deep brain stimulation for Parkinson's disease. Stereotact Funct Neurosurg. (2013) 91:12–7. doi: 10.1159/000342161, PMID: 23154788

[9] LjungHNordlundAStrandbergMBengzonJKällénK. Verbal memory decline from hippocampal depth electrodes in temporal lobe surgery for epilepsy. Epilepsia. (2017) 58:2143–52. doi: 10.1111/epi.13931, PMID: 29105058

